# Changes in Physical Health-Related Indexes of Chinese College Students before and after COVID-19 Lockdown

**DOI:** 10.1155/2022/7802492

**Published:** 2022-08-16

**Authors:** Donglin Hu, Zhiyun Liu, He Zhang, Chen Jiang

**Affiliations:** ^1^Department of Physical Education, Nanjing Agricultural University, Nanjing, China; ^2^Tianjin University of Sport, Tianjin, China; ^3^Faculty of Health, Southern Cross University, Lismore, New South Wales, Australia; ^4^Department of Physical Education, Nanjing Audit University, China

## Abstract

The outbreak of the COVID-19 pandemic has caused negative impacts on people's lifestyles, as well as considerable indirect social impacts, which has even overshadowed the direct impact of virus infection itself. This study is aimed at examining the changes in physical health-related indexes of Chinese college students before and after the COVID-19 lockdown. The data of this study are from the National Physical Health Testing Program, covering 43 college students (male: 22) from a class of a Chinese university. Paired *t*-tests were performed on the physical health test data separately collected in November 2019 before the COVID-19 pandemic and October 2020 after the COVID-19 lockdown was lifted. As shown by the test results, compared to the prelockdown data, college students had an increased body mass index (BMI) (0.43 (SD 0.94) *P* = 0.004), decreased vital capacity (VC) (-128.98 (SD 310.13) ml *P* = 0.009), and lowered performance in the 800/1000 m endurance (-6.21 (SD 8.81) points *P* < 0.001) and standing long jump tests (-2.44 (SD 7.37) points *P* = 0.036) after the lockdown, and the differences in these regards all were significant. In addition, for the students in the overweight/obese group, their pre- and postlockdown physical fitness test results were found to have no statistically significant difference (*P* > 0.05), but the students in the control group showed a significantly increased BMI, as well as significantly decreased vital capacity and performance in the 800/1000 m endurance and standing long jump tests (*P* < 0.05). The findings of this study are expected to help government departments and policymakers better understand the impacts of school closures and online learning on the physical health of adolescents, while providing a basis for the formulation of measures that are aimed at reversing adolescents' physical health decline.

## 1. Introduction

The coronavirus disease 2019 (COVID-19) was first identified in 2019 and then spread to most countries around the world within just a few months [1]. On 30 January 2020, the World Health Organization (WHO) declared the pandemic a Public Health Emergency of International Concern. As of October 22, 2021, the pandemic situation remains severe, with more than 200 countries and regions around the world affected and 242,348,657 confirmed cases, of which 4,927,723 were dead [2]. The pandemic has caused huge negative impacts on society, economy, and life worldwide and seriously threatened people's lives. In response, governments around the world, especially the Chinese government, have implemented a series of drastic measures, such as partial lockdown and social isolation, closing schools, factories, and nonessential public places. These measures have effectively reduced cross infection to varying degrees.

One of the most important responsive policies taken by the Chinese government was to close schools and launch online teaching as an alternative. Although social distancing and lockdown policies are effective measures to contain the spread of the pandemic, they have dramatically changed the lifestyles of the public. Additionally, prolonged online learning and school closures have caused another unexpected consequence, that is, the sharp decline of children and adolescents in physical activity and the increased risk of their physical and mental health as a result [1]. Physical activity is defined as any physical movement of skeletal muscle that consumes energy [3]. For children and adolescents, physical activity includes play, games, sports, transportation, recreation, physical education, or planned exercise in the context of family, school, and community activities. Physical inactivity may produce a series of health risks, including high cholesterol, elevated blood pressure, and increased risk of diabetes [4, 5]. The purpose of this study is to identify the changes in physical health-related indexes of Chinese college students before and after the COVID-19 lockdown.

## 2. Research Methods

### 2.1. Research Design

The research data came from Physical Activity and Fitness in China (PAFC), a physical fitness testing program for children and adolescents initiated by the Ministry of Education of China, which examined and assessed the physical fitness of school-age children and adolescents nationwide at the beginning of each academic year (September-November) using a cross-sectional design. This study is part of the program, focusing on the testing of adolescents in colleges and universities with the items specified in the 2014 National Standards for Physical Fitness. The test items can be classified into six parts: BMI, seated forward bends (flexibility), standing long jump (explosive strength), sit-ups for girls (abdominal muscle strength), pull-ups for boys (upper body muscle strength), 1000 m race for boys/800 m race for girls (cardiorespiratory endurance), and vital capacity (cardiorespiratory function). The subjects were from a university in China, and the test was conducted at a uniform time and place to maintain the consistency by physical education teachers of the university who received professional training and had rich experience.

With the paired *t*-test method, this study compared the physical health test data in November 2019 before the COVID-19 pandemic and October 2020 after the release of school lockdown, with the aim of exploring the changes in physical health-related indexes such as BMI before and after school closure.

This study protocol was approved by the Ethics Review Committee of Tianjin University of Sport, and the teachers and principal of the surveyed school granted their consent. In addition, all participating students were informed of the content and purpose of this study and granted their informed consent orally before the data were collected. The data were collected anonymously and then stored in an encrypted hard disk.

### 2.2. Participants

The participants in this study were 43 students from the same class at a Chinese university, including 22 males and 21 females. All of them were Han Chinese, in good health with no disabilities. The first test was performed before the COVID-19 outbreak (November 2019), and the data collected would be used as the benchmark. After the pandemic was controlled in China and offline teaching was resumed (October 2020), the second test was conducted. This study longitudinally compared the test data in November 2019 and October 2020. The difference in BMI between male and female students was insignificant (*P* > 0.05), but the height and weight of male students were significantly higher than female ones (*P* < 0.05), as shown in Table 1.

### 2.3. Data Analysis

A paired *t*-test was used to assess the changes in the physical fitness of college students before the lockdown (November 2019) and after it was lifted (October 2020). Pearson correlation analysis was utilized to identify the relations before and after COVID-19 lockdown in terms of BMI, flexibility, muscle strength, cardiopulmonary function, and cardiopulmonary endurance. All analyses were performed using Statistical Package or the Social Sciences Version 26.0 (SPSS Inc., Chicago, IL), and a bilateral *P* value of less than 0.05 was considered statistically significant.

### 2.4. Data Collection

The items specified in the 2014 National Student Physical Health Standards were used for physical fitness assessment. The items fall into five tests to measure different health dimensions, including BMI, seated forward bends, standing long jump, sit-ups for girls, pull-ups for boys, and 1000 m race for boys/800 m race for girls.

#### 2.4.1. BMI

The height and weight of students barefoot and wearing light clothes were measured using an integrated intelligent measuring device (Hongtai S150, Shanghai), with the values correct to 0.01 m and 0.1 kg, respectively. BMI is calculated by dividing a student's weight by the square of his/her height (BMI = weight (kg)/height (m^2^)). The data on height and weight were collected in a quiet room to protect personal privacy.

#### 2.4.2. Cardiorespiratory Endurance

Cardiorespiratory endurance was assessed by a 1000 m race for boys and an 800 m race for girls. The races were conducted in a standard sports field on the university campus, and the students were asked to complete the race as quickly as possible while maintaining a steady pace. An electronic stopwatch was for timekeeping (XINJIE XJ-894, Jinhua, China). During the measurement, physical education teachers were responsible for race safety and quality supervision.

#### 2.4.3. Cardiopulmonary Function

The cardiopulmonary function of college students was represented by their vital capacity, which was measured and recorded by physical education teachers using a digital spirometer (WQS-8888, Beijing).

#### 2.4.4. Flexibility

The value was measured and recorded by physical education teachers using a seated forward bending tester (ZWTQQ-007, Jinhua, China) that could be correct to 0.1 cm.

#### 2.4.5. Strength Quality

Items including standing long jump, 50 m sprint, pull-ups for boys, and sit-ups for girls were carried out for assessment. Standing long jump and 50 m sprint have been widely applied to explosive strength assessment. Pull-ups for boys had no time limit and were used to assess upper body strength, while sit-ups for girls were used to assess abdominal strength, with a time limit of 1 minute. All the test items were conducted under the supervision of physical education teachers, who were also responsible for the safety.

All the aforesaid test items were given a final score in the range of 0-100 according to the National Student Physical Health Standards (2014 Edition).

## 3. Results

The variables including BMI, vital capacity, cardiorespiratory endurance, flexibility, and strength quality were denoted as mean ± standard deviation (SD). All variables were normally distributed (see Table 2). Paired *t*-tests were carried out to compare the differences in physical health indexes of college students before and after the pandemic (see Table 3). The *P* values in the 50 m sprint, pull-ups/sit-ups test, and flexibility test were 0.098, 0.064, and 0.982, respectively, all exceeding 0.05, so the differences had no statistical significance. The BMI was found to have significantly increased after the lockdown was lifted (0.64 (SD 1.46) *P* = 0.006). The vital capacity decreased significantly compared with the time before the pandemic (-128.98 (SD 310.13) ml *P* = 0.009), so did the scores of the 800/1000 m endurance races (-7.19 (SD 10.16) *P* < 0.001). The scores of standing long jump were lower than the time before the pandemic (-2.44 (SD 7.37) *P* = 0.036) as well, and the difference was statistically significant.

With the prepandemic physical fitness test data as the benchmark, the subjects were classified into an overweight/obese group (BMI ≥ 24) and a normal-weight control group (BMI < 24) according to the BMI reference norm for screening overweight and obesity in Chinese children and adolescents [6]. The results showed that for the students in the overweight/obese group, the pre- and postlockdown physical fitness test results were not statistically significantly different (*P* > 0.05); but for the students in the control group, they experienced an increased BMI, decreased vital capacity and cardiorespiratory endurance, and worse performance in standing long jump, and the differences were statistically significant (*P* < 0.05), as shown in Table 4.

## 4. Discussion

This study is part of the research on the effects of school closures on the BMI, muscle strength, cardiopulmonary function, and flexibility of adolescents during the COVID-19 pandemic. In this study, all participants performed 15-18 weeks of online learning, and paired *t*-tests were conducted to compare the physical health data (benchmark data) before the pandemic and those after the lockdown. It was found that the *P* values of BMI, vital capacity, endurance quality, and standing long jump were all less than 0.05, and the difference was statistically significant. However, the *P* values of pull-ups/sit-ups, flexibility, and 50 m race exceeded 0.05, and the difference was not statistically significant.

The results revealed that after social isolation and school closures, college students had significantly increased BMI and decreased vital capacity, endurance, and strength quality, suggesting that online learning in the months of the pandemic lockdown may affect adolescents' health-related indexes. This finding is consistent with the results of previous studies [7–10], which concluded that decreased physical activity and increased sedentary behavior in children and young people affected their physical health indexes.

Additionally, the results of this study showed that college students' BMI increased by 0.43 ± 0.94 (0.14(0.72) 95% CI) after the lockdown was lifted, which was atypical compared with the situation reported before COVID-19. This is because the BMI of children and young people is usually controlled during the school year. Previous studies have shown that among college students, BMI would slightly drop during the school year [11–13].

The increased BMI found in this study is not surprising given school closures, cancellation of sports activities, and sedentary lifestyles due to long-time online learning. Although such an analysis must be performed prudently, the rise of BMI is probably due to the month-long online learning and social isolation. At present, some areas of China are still subject to social isolation and school lockdown, which may prompt the reuse of online teaching in some schools in the future. Therefore, it is of great necessity to create safe and continuous physical activity opportunities for young people, in an effort to prevent students from physical inactivity.

In addition, this study found that for the students in the overweight/obese group (BMI ≥ 24), the difference between pre- and postlockdown performance in the tests was statistically insignificant (*P* > 0.05), but for the students in the control group (BMI < 24), their pre- and postlockdown performance in BMI, vital capacity, cardiorespiratory endurance, and standing long jump were all significantly different (*P* < 0.05). Contrary to the conclusion that overweight/obese children were more likely to be affected by schooling suspension or school closure [14], the insignificant differences are probably attributed to the smaller influence of school closure and physical activity cancellation on overweight/obese college students who generally prefer to a sedentary lifestyle. In contrast, for the students in the control group (BMI < 24), the lockdown or social distancing has heavily affected their daily life, resulting in their significantly reduced physical health levels, such as an increased BMI, decreased vital capacity and cardiorespiratory endurance, and lowered performance in the standing long jump. These results were worrisome since their performance in those aspects was supposed to be improved with the progress of the academic year [15–18]. These findings implied that the adolescents participating in this study were largely inactive, as could be seen from the sharp decline in cardiopulmonary endurance, which also proved the considerable impact of online learning and school closures on college students. Therefore, government departments or policymakers should pay sufficient attention to this problem and develop countermeasures to reverse the continued decline. In particular, it is possible to see repeated pandemic outbreaks in the future and resultant school closures that lead to online teaching necessary. Therefore, it is imperative for relevant departments to take action.

This study also has several limitations. First of all, the sample size was small (*N* = 43), and the participants were only the students of one class in a Chinese university. Hence, the sample size in future research needs to be expanded. Besides, some variables that might affect the results are not taken into account, such as dietary habits, sleep quality, and living habits like smoking and drinking.

Moreover, since Chinese universities had resumed offline teaching in September 2020, September rather than October may be the most ideal month for the second test.

## 5. Conclusion

In summary, the indirect impact of the COVID-19 pandemic has exceeded the impact caused by the virus infection itself. Measures taken against the pandemic such as social isolation and school closures have adversely affected the healthy lifestyle of people. However, having a clear understanding of the consequences brought about by lockdown is just the first step to taking preventive measures. This study provides preliminary data about the impact of COVID-19 lockdown on the physical fitness of Chinese college students. To the best of our knowledge, it is the first longitudinal study exploring the changes in the physical fitness of Chinese college students in the context of COVID-19. This study sheds new insights into the future exploration of the impact of school closures or online learning on the physical fitness of children and adolescents, and its findings are expected to provide a reference for government departments and policymakers to formulate countermeasures that are aimed at enhancing young people's health.

## Figures and Tables

**Table 1:** Descriptive characteristics of study subjects.

Sex	Number of participants	Age (Y) *M* ± SD	Height (m) *M* ± SD	Weight (kg) *M* ± SD	BMI *M* ± SD
Males	22	20.27 ± 0.70	1.78 ± 0.52	73.40 ± 18.01	23.17 ± 5.07
Females	21	20.33 ± 0.48	1.63 ± 0.06	55.42 ± 8.19	20.76 ± 2.37
*t*		-0.328	8.37	4.25	1.98
*P*		0.745	<0.001	<0.001	0.054

Notes: BMI: body mass index; *M* ± SD: mean ± standard deviation.

**Table 2:** Tests of normality.

	Kolmogorov-Smirnov			Shapiro-Wilk		
	Statistic	df	Sig.	Statistic	df	Sig.
*Δ*1	.068	43	.200	.982	43	.744
*Δ*2	.121	43	.116	.958	43	.112
*Δ*3	.090	43	.200^∗^	.984	43	.803
*Δ*4	.137	43	.040	.962	43	.159
*Δ*5	.126	43	.082	.964	43	.190
*Δ*6	.119	43	.134	.953	43	.079
*Δ*7	.130	43	.065	.968	43	.276

Notes: *Δ*: lockdown lifted-baseline value, pairing differences; *Δ*1: BMI; *Δ*2: vital capacity; *Δ*3: 50 m sprint; *Δ*4: 800/1000 m; *Δ*5: standing long jump; *Δ*6: flexibility; *Δ*7: strength.

**Table 3:** Paired samples test.

Variable	Baseline	Lockdown lifted	*Δ*	95% CI	*t*	*P*
BMI	21.99 ± 4.12	22.43 ± 4.14	0.43 ± 0.94	0.14 (0.72)	3.02	0.004^∗∗^
Vital capacity	4230.23 ± 1379.18	4101.26 ± 1288.73	-128.98 ± 310.13	-224.42(-33.53)	-2.73	0.009^∗∗^
50 m Sprint	72.65 ± 8.30	71.02 ± 7.53	−1.63 ± 6.32	-3.57 (0.32)	-1.69	0.098
800/1000 m	70.93 ± 6.77	64.72 ± 9.36	−6.21 ± 8.81	-8.92(-3.50)	-4.62	<0.001^∗∗^
Strength	45.33 ± 34.55	44.79 ± 33.87	−0.537 ± 1.85	-1.11 (0.033)	-1.90	0.064
SLG	72.72 ± 9.44	70.28 ± 8.72	−2.44 ± 7.37	-4.71(-1.73)	-2.17	0.036^∗^
Flexibility	75.30 ± 11.21	75.28 ± 9.12	−0.23 ± 6.68	-2.08 (2.03)	-0.23	0.982

Notes: *N* = 43; SLG: standing long jump; ^∗^*P* < .05; ^∗∗^*P* < .01; *Δ*: lockdown lifted-baseline value.

**Table 4:** Paired samples test.

Participants	Time	*S*	BMI	VC	50 m	800/1000 m	Strength	SLG	Flexibility
Overweight/obese	Baseline		29.00 ± 3.10	5442.63 ± 1548.24	71.25 ± 5.75	62.25 ± 5.55	45.50 ± 41.55	64.75 ± 2.27	76.50 ± 7.15
	Lockdown lifted		29.45 ± 2.79	5417.63 ± 1499.80	70.63 ± 8.23	60.13 ± 8.39	44.88 ± 41.47	66.88 ± 2.86	77.13 ± 4.88
		*Δ*	0.45 ± 0.94	25.00 ± 336.96	0.63 ± 4.93	5.13 ± 7.77	0.63 ± 1.92	−2.13 ± 5.91	−0.63 ± 5.78
		*t*	-1.37	0.21	0.36	1.87	0.919	-1.02	-0.31
		*P*	0.215	0.840	0.730	0.104	0.388	0.343	0.769

Control group	Baseline		20.39 ± 2.19	3953.11 ± 1196.36	72.97 ± 8.82	72.23 ± 6.39	45.29 ± 33.45	74.54 ± 9.12	75.03 ± 12.02
	Lockdown lifted		20.82 ± 2.30	3800.37 ± 1042.87	71.11 ± 7.49	65.77 ± 9.36	44.77 ± 32.60	71.06 ± 8.78	74.86 ± 9.84
		*Δ*	−4.23 ± 0.95	152.74 ± 303.83	1.86 ± 6.63	6.46 ± 9.11	0.52 ± 1.86	3.49 ± 7.34	0.17 ± 6.94
		*t*	-2.66	2.97	1.66	4.191	1.642	2.81	0.146
		*P*	0.012^∗^	0.005^∗∗^	0.107	<0.001^∗∗^	0.110	0.008^∗∗^	0.885

Notes: *S*: statistic; VC: vital capacity; 50 m: 50 m sprint; SLG: standing long jump; ^∗^*P* < .05; ^∗∗^*P* < .01; *Δ*: lockdown lifted-baseline value.

## Data Availability

Requests for access to individual subject data may be made to Donglin Hu; please send an email to 2011022@njau.edu.cn.
